# Programmed death-ligand 1 is upregulated in intrahepatic lymphoepithelioma-like cholangiocarcinoma

**DOI:** 10.18632/oncotarget.11949

**Published:** 2016-09-10

**Authors:** Lei Wang, Hui Dong, Shujuan Ni, Dan Huang, Cong Tan, Bin Chang, Weiqi Sheng

**Affiliations:** ^1^ Department of Pathology, Fudan University Shanghai Cancer Center, Shanghai, 200032, China; ^2^ Department of Oncology, Shanghai Medical College, Fudan University, Shanghai, 200032, China; ^3^ Department of Pathology, Shanghai Eastern Hepatobiliary Surgery Hospital, The Second Military Medical University, Shanghai, 200438, China

**Keywords:** intrahepatic cholangiocarcinoma, intrahepatic lymphoepithelioma-like cholangiocarcinoma, clinicopathological characteristics, PD-L1, clinical outcomes

## Abstract

Intrahepatic lymphoepithelioma-like cholangiocarcinoma (LELCC) is a rare variant of cholangiocarcinoma. Here, we report the largest single series of LELCC cases yet studied (*n* = 13). We retrospectively analyzed the clinical data of the 13 patients and measured the expression of programmed death-ligand 1 (PD-L1) in tumors using immunohistochemical staining. We also analyzed 15 cases of conventional intrahepatic cholangiocarcinoma (IHCC) for comparison. We found that eight patients with LELCC were infected with Epstein-Barr Virus (EBV), and EBV infection correlated with poor prognosis in LELCC. Four patients among the five (80.0%) without EBV had a history of chronic viral hepatitis B. None of the 15 cases of conventional cholangiocarcinoma were positive for EBV. PD-L1 was expressed in both the tumor cells and tumor-infiltrating immune cells in LELCC patients at higher levels than in IHCC patients (*P* < 0.05). These observations suggest that EBV infection may promote the development of LELCC, and that PD-L1 may be a potential therapeutic target for treatment of EBV-associated LELCC.

## INTRODUCTION

Lymphoepithelioma-like carcinomas (LELCs) are tumors characterized by undifferentiated carcinomas with prominent tumor-infiltrating lymphocytes (TILs) identical to undifferentiated nasopharyngeal carcinoma (NPC). LELCs have been reported in multiple human organs and different types of human tissue [1–7]. Lymphoepithelioma-like cholangiocarcinoma (LELCC), a form of LELC that develops from the hepatobiliary tract, is a rare variant of intrahepatic cholangiocarcinoma. Because of the limited number of cases reported (only 26 in the literature in English [8–23]), further research is needed to better characterize the clinicopathological features of LELCC.

Cytotoxic tumor-infiltrating lymphocytes help eliminate cancer cells and prevent recurrence. However, cancer cells can escape immune surveillance. Programmed death-1 (PD-1) is an immunosuppressive receptor expressed in active T cells [24, 25] that has been found in TILs in several types of cancer [26–29]. Programmed death-ligand 1 (PD-L1) is a PD-1 ligand that is expressed in tumor cells, some immune cells [30], and some virus-associated malignancies [31]. In EBV-positive NPC cell lines, expression of PD-L1 was higher compared with controls [32]. In LELCC, 73.1% (19/26) of reported cases were associated with EBV infection. In this study, to better understand the clinicopathological features of LELCC, we analyzed 13 new cases, measuring the expression pattern of PD-L1 and analyzing the relationship between EBV infection and PD-L1 expression.

## RESULTS

Sixteen studies describing a total of 26 cases of LELCC have been reported [8–23]. In this study, we analyzed 13 additional cases (the largest single series reported to date). Among a total of 39 cases of LELCC, 89.7% (35/39) were from Asia (China 14/35, 40.0%; Taiwan 9/35, 25.7%; Hong Kong 7/35, 20.0%; Korea 3/35, 8.6%; Japan 2/35, 5.7%). Slight female preponderance was observed (22 females and 17 males). The mean and median ages were 54.4 and 57 years (range 19–78 years).

### Clinical data

All patients in our 13-case cohort underwent extensive systemic examination preoperatively, and all were negative for tumors other than liver tumors. The clinical features of LELCC and IHCC are summarized in Tables 1 and 2. The mean and median age of LELCC patients was 53.5 and 53.0 years (range 35–71 years) and the male/female ratio was 2.3:1. The mean and median age of IHCC patients was 61.1 and 58.0 years (range 41–77 years) and the male/female ratio was 2.8:1. Six LELCC patients (6/13, 46.2%) and only one IHCC patient (1/15, 6.7%) had a history of chronic viral hepatitis B (HBV), while none of them had a history of chronic viral hepatitis C (HCV). The median follow-up intervals of LELCC patients and IHCC patients were 22 months (ranging from 8 to 54 months) and 18 months (ranging from 10 to 40 months), respectively. The disease-specific survival (DSS) rate at three years was 72.0% for LELCC and 34.0% for IHCC, but the difference was not statistically significant (*P* = 0.089) (Figure 1). At the end of the follow-up period (a median follow-up interval of 27 months, ranging from 8 to 54 months), 10 LELCC patients (76.9%) were alive with no evidence of disease while one LELCC patient (7.7%) developed local recurrence 10 months after surgery. Two LELCC patients (15.4%) died of the disease at 27 and 22 months after the surgery. On the other hand, only three IHCC patients (20.0%) were alive without the disease at the end of the follow-up period (median interval of 17 months, ranging from 11 to 25 months), and seven IHCC patients (46.7%) died of the disease.

**Table 1:** Clinical characteristic of lymphoepithelioma-like cholangiocarcinoma

Case	Age (year)	Sex	Tumor site	Tumor size (cm)	HBV	HCV	EBER	AFP (ng/ml)	CA199 (u/ml)	Clinical outcome
1	60	M	Right lobe	6.0	+	−	+	2.1	1.1	DOD, 27 months follow-up
2	53	M	Right lobe	2.4	−	−	+	2.7	23.1	DOD, 22 months follow-up
3	39	M	Left lobe	2.0	−	−	−	3.0	7.6	AWOD, 54 months follow-up
4	43	F	Right lobe	1.2	−	−	+	2.3	7.4	AWOD, 51 months follow-up
5	62	M	Right lobe	3.2	+	−	−	4.7	36.0	AWOD, 37 months follow-up
6	65	F	Right lobe	5.0	+	−	−	42.4	21.0	AWOD, 37 months follow-up
7	47	F	Left lobe	1.9	−	−	+	1.9	2.7	AWOD, 35 months follow-up
8	52	M	Right lobe	1.9	+	−	−	1.3	9.8	AWOD, 19 months follow-up
9	60	M	Left lobe	2.6	−	−	+	1.5	15.5	AWOD, 12 months follow-up
10	61	M	Right lobe	2.4	+	−	−	3.8	14.7	AWD, 12 months follow-up Intrahepatic recurrence (10 months)
11	35	M	Right lobe	3.1	+	−	+	3.3	13.1	AWOD, 10 months follow-up
12	48	M	Right lobe	3.5	−	−	+	1.4	3.5	AWOD, 9 months follow-up
13	71	F	Right lobe	2.2	−	−	+	1.7	4.0	AWOD, 8 months follow-up

AWOD, Alive without disease; AWD, alive with disease; DOD, died of disease.

**Table 2:** The summary of clinical characteristic of intrahepatic cholangiocarcinoma (IHCC) and intrahepatic lymphoepithelioma-like cholangiocarcinoma (LELCC)

	LELCC (*n* = 13)	IHCC (*n*= 15)	*P*
Age (years)	53.5 ± 3.0	61.1 ± 3.0	0.674
Mean age	53.5	61.1	
Median age	53.0	58.0	
Sex			0.814
Female (%)	4 (30.8%)	4 (26.7%)	
Male (%)	9 (69.2%)	11 (73.3%)	
Tumor site			0.053
Left lobe (%)	3	9	
Right lobe (%)	10	6	
Tumor size (cm)	2.9 ± 0.4	5.5 ± 0.6	0.067
Mean size	2.9	5.5.	
Median size	2.4	5.0	
HBV			0.018
Positive (%)	6 (46.2%)	1 (6.7%)	
Negative (%)	7 (53.8%)	11 (93.3%)	
HCV			
Positive (%)	0	0	
Negative (%)	13 (100%)	15 (100%)	
EBV			< 0.001
Positive (%)	8 (61.5%)	0	
Negative (%)	5 (38.5%)	15 (100%)	
Median follow-up period (months)	22	18	
Disease-specific survival			
3-year (%)	72.0%	34.0%	0.089

**Figure 1:** Kaplan-Meier disease-specific survival curves for intrahepatic lymphoepithelioma-like cholangiocarcinoma (LELCC) and conventional intrahepatic cholangiocarcinoma (IHCC)

### Pathological findings

In our cohort, 10 LELCC tumors (76.9%) were located in the right hepatic lobe, while nine IHCC tumors (60.0%) were located in the left lobe (*P* = 0.053). The size of LELCC tumors ranged from 1.2 to 6.0 cm in diameter (mean, 2.9 cm; median, 2.4 cm), which was smaller than that of IHCC tumors (mean, 5.5 cm; median, 5.0 cm) (*P* = 0.067). The pathological features are shown in Table 3. Histologically, a lymphoepithelioma pattern can be observed in all cases. There were two components: 1) sheets of large tumor cells with vesicular nuclei, prominent nucleoli, and a syncytial cytoplasmic appearance (lymphoepithelioma-like carcinoma component) (Figure 2A), and 2) glandular differentiation (adenocarcinoma component) (Figure 2B). Both components were merged together and with a dense lymphocytic infiltration component. The adenocarcinoma component can be further divided into with and without an intense lymphocytic infiltration. As shown in Table 3, the proportions of lymphoepithelioma-like carcinoma component and of adenocarcinoma component with and without an intense lymphocytic infiltration were calculated for every case, separately. There were five cases (38.5%) showing lymphoepithelioma-like carcinoma as a predominant component (≥ 90%). Different from conventional IHCC, significant desmoplasia was not observed in LELCC, even in the adenocarcinoma component.

**Table 3:** Histological and immunohistochemical characteristics of lymphoepithelioma-like cholangiocarcinoma

Case	LELC Component	GCWLI	GCWOLI	HepPar−1	CK7	CK19	PD−L1		EBER
							Tumor cells	Immune cells	
1	60%	40%	0	−	+	+	−	+ (2)	+
2	80%	20%	0	−	+	+	+ (3)	+ (2)	+
3	90%	10%	0	−	+	+	+ (3)	+ (1)	−
4	> 90%	< 10%	0	−	+	+	−	+ (3)	+
5	> 90%	< 10%	0	−	+	+	+ (3)	+ (2)	−
6	80%	0	20%	−	+	+	+ (3)	+ (2)	−
7	40%	60%	0	−	+	+	−	+ (3)	+
8	90%	10%	0	−	+	+	+ (1)	+ (2)	−
9	60%	40%	0	−	+	+	+ (1)	+ (1)	+
10	70%	30%	0	−	+	+	+ (1)	+ (2)	−
11	90%	10%	0	−	+	+	+ (1)	+ (1)	+
12	60%	40%	0	−	+	+	+ (1)	+ (2)	+
13	80%	20%	0	−	+	+	+ (2)	+ (2)	+

LELC, lymphoepithelioma-like carcinoma.

GCWLI, Glandular component with lymphocytic infiltration.

GCWOLI, Glandular component without lymphocytic infiltration.

The negative cases ‘−’ < 5% positive.

The intensity of PD-L1 expression was scored as follows: 1, weak; 2, moderate; and 3, strong staining in more than 5% of cells.

**Figure 2:** Histological features of lymphoepithelioma-like cholangiocarcinoma (**A**) The lymphoepithelioma-like carcinoma component consisted of sheets of large tumor cells with a syncytial cytoplasmic appearance and dense lymphocytic infiltration. (**B**) The adenocarcinoma component consisted of irregular malignant glands with dense lymphocytic infiltration. (**C**) The nuclei of tumor cells, but not the tumor-infiltrated immune cells, were positive for EBER. HE, ×400.

EBER was positive in the nucleus of tumor cells in the adenocarcinoma and lymphoepithelioma-like carcinoma components of eight LELCC cases (8/13, 61.5%) (Figure 2C), but not in tumor-infiltrated immune cells. EBER was negative in all 15 cases of IHCC. As shown in Table 1, six of the eight (75.0%) EBV-positive LELCC patients were not infected by HBV, while four of the five (80.0%) LELCC patients without EBV infection had a history of chronic viral hepatitis B. Ten LELCC patients (76.9%) were infected with EBV or HBV. Three of five cases (60.0%) showing lymphoepithelioma-like carcinoma as a predominant component (≥ 90%) were EBER negative while among the other eight cases showing a higher proportion of adenocarcinoma component only two cases (25.0%) were EBER negative (*P* = 0.249) (Table 3). Two patients who died of the disease were EBER positive. Taking into account the cases of LELCC reported previously in the literature, among a total of 39 LELCC patients, only five (12.8%) died of the disease and were infected by EBV. Patients without EBV infection appeared to survive longer than EBER positive patients (Figure 3); however, the differences between these two groups were not significant (*P* = 0.161) because of the small sample size.

**Figure 3:** Kaplan-Meier disease-specific survival curves for patients with and without EBV infection

### Immunohistochemical features

The results of immunohistochemical staining are summarized in Tables 3 and 4. The adenocarcinoma component of the LELCC was diffusely positive for CK7 and CK19, while the lymphoepithelioma-like carcinoma component was focally positive for CK7 and CK19 in some cases (Figure 4A–4D). All cases were negative for HepPar-1 (Figure 4E). PD-L1 was detected in tumor cells and/or tumor-infiltrating immune cells with variable intensities and proportions (Figure 5). PD-L1 expression in tumor cells was observed in 76.9% (10/13) of LELCC and 26.7% (4/15) of IHCC (*P* = 0.011). On the other hand, for tumor-infiltrating immune cells, PD-L1 was positive in 100.0% (13/13) of LELCC and 20.0% (3/15) of IHCC cases (*P* < 0.001) (Table 4). In 10 cases with PD-L1 positive tumor cells, six cases (case 2, 3, 5, 8, 12, 13) expressed PD-L1 both in the lymphoepithelioma-like carcinoma and glandular component. PD-L1 expression was observed only in the lymphoepithelioma-like carcinoma component in four cases (case 6, 9, 10, 11). Of the eight cases with EBV infection, five expressed PD-L1 in tumor cells while the other three were PD-L1 negative. All 5 cases without EBV infection expressed PD-L1 (*P* = 0.134). In all cases (13 cases of LELCC and 15 cases of IHCC), PD-L1 expression in tumor-infiltrating immune cells was higher in the patients with EBV infection (*P* = 0.004) (Table 5). PD-L1 expression was also more common in tumor cells from patients with EBV infection (62.5%) than in those from patients without EBV infection (45.0%), but the difference was not statistically significant (*P* = 0.339) (Table 5).

**Table 4:** PD-L1 expression in intrahepatic lympoeithelioma-like cholangiocarcinoma (LELCC) and intrahepatic cholangiocarcinoma (IHCC)

	LELCC (*n*= 13)	IHCC (*n* = 15)	*P*
PD-L1 expression in tumor cells			0.011
+	10	4	
−	3	11	
PD-L1 expression in immune cells			< 0.001
+	13	3	
−	0	12	
EBER			< 0.001
+	8	0	
−	5	15	

**Figure 4:** Immunohistochemical features of lymphoepithelioma-like cholangiocarcinoma The adenocarcinoma component is diffusely positive for (**A**) CK7 and (**B**) CK19, while the lymphoepithelioma-like carcinoma component is focally positive for (**C**) CK7 and (**D**) CK19. (**E**) The tumor cells of both components were negative for HepPar-1. Immunohistochemistry, ×200.

**Figure 5:** Representative images of PD-L1 immunostaining PD-L1 was immunostained on the membrane and/or in the cytoplasm of tumor cells with variable intensities: (**A**–**D**) absent in the conventional IHCC (score 0), weak in LELCC (score 1), moderate in LELCC (score 2), strong in LELCC (score 3). In most cases, PD-L1 was expressed in tumor cells, which were highlighted by (**E**) AE1/AE3, and (**F**) tumor-infiltrated immune cells. (**H**) In 3 cases, PD-L1 was immunostained mainly in tumor-infiltrated immune cells, (**G**) with little staining in tumor cells, which were highlighted by AE1/AE3. Immunohistochemistry, ×200.

**Table 5:** The relationship between PD-L1 expression and EBV infection in all the cases of cholangiocarcinoma

	EBER		*P*
	+ (*n* = 8)	− (*n* = 20)	
PD-L1 expression in tumor cells			0.339
+	5	9	
−	3	11	
PD-L1 expression in immune cells			0.004
+	8	8	
−	0	12	

## DISCUSSION

Lymphoepithelioma-like cholangiocarcinoma is a rare variant of IHCC, displaying distinct clinicopathological characteristics. Unlike lymphoepithelioma-like carcinomas (LELCs) of organs other than the liver, the majority of LELCCs have two different components–the adenocarcinoma component and the lymphoepithelioma-like carcinoma component, both of which were merged together for our analyses in this study. Glandular differentiation is a diagnostic hallmark of LELCC; however, there are two reported cases without glandular differentiation [15, 17]. On the contrary, it is common for LELC of organs other to not present glandular differentiation. Lymphoepithelioma-like carcinoma has also been reported in the extrahepatic bile duct. There is only one case (also from Asia) of LELC of the inferior common bile duct reported in the literature in English [33]. Histologically, the tumor contained lymphoepithelioma-like carcinoma and adenocarcinoma components, similar to LELCC. The major differential diagnosis was lymphoepithelioma-like hepatocellular carcinomas (LEL-HCC), also a rare variant of HCC [34], and metastatic LELCs from other sites. However, additional studies and more cases are needed to better characterize the clinicopathological features of extrahepatic LELCC.

LELCs are usually associated with EBV [35]. EBV integration was found in 19 cases (73.1%) among the previously reported 26 cases. In our cohort, 8 out of 13 cases (61.5%) presented EBV infection. On the other hand, none of the 15 cases of conventional cholangiocarcinoma were positive for EBV. These results suggest that EBV infection might promote the development of LELCC. The majority cases of LELCC were from South China and Taiwan, where EBV is prevalent [36]. Seven of the 26 previously reported cases of LELCC were negative for EBV, with one presenting HCV infection and two presenting HBV infection. In our cohort, 4 of the 5 EBV negative patients had HBV infection. These findings suggest that HBV and HCV may also promote the development of LELCC.

We found that the clinical outcome of LELCC is more favorable than that of conventional cholangiocarcinoma. Also, although a better prognosis can be observed in patients with EBV-associated malignancies in stomach [37] and lung [38] LELC, among all previously reported cases of LELCC combined, only 5 patients (14.7%) died of the disease, all of which were positive for EBV. This suggests that EBV infection leads to poorer prognosis in LELCC. However, because of the rarity of LELCC, further studies are needed to confirm the correlation between EBV infection status and prognosis.

The immune regulatory PD-L1/PD-1 axis, which protects the host from overactive T-cells, may play an important role in the progression of virus associated malignancies [39, 40]. Therefore, the PD-L1/PD-1 axis can be targeted by immunotherapy against virus-associated cancer. However, the identification of predictive markers for effective immunotherapy remains challenging. In early clinical trials, PD-L1 expression in tumor cells was used as a biomarker for selecting patients for PD-1/PD-L1 inhibitor therapy. Importantly, positive PD-L1 tumor expression was correlated with higher response rates in many types of tumors. However, many PD-L1 negative patients also experienced benefits from PD-1/PD-L1 inhibitor treatment [41]. Herbst *et al.* [42] observed a positive response to anti-PD-L1 antibody in patients with high levels of PD-L1 suffering from various types of cancer, especially when PD-L1 was expressed in immune cells. Recent studies [43, 44] highlight PD-L1 expression as a candidate marker for immunotherapy with anti-PD-1 antibody.

In our study, we measured PD-L1 expression in LELCC and conventional IHCC. We found that while PD-L1 was expressed in tumor cells and tumor-infiltrating immune cells in both LELCC and IHCC, PD-L1 levels were higher in LELCC than in IHCC. Similar results were previously reported for EBV-infected nasopharyngeal carcinoma (NPC) [32], EBV-related B-cell lymphoma [31], and EBV-positive Hodgkin lymphoma [45]. These findings indicated that the chronic inflammatory environments of virus-associated cancers may promote PD-L1 upregulation. Therefore, PD-L1/PD-1 may be targeted with therapeutic benefits in EBV-associated malignancies. Recently, Fang *et al.* [32] investigated the mechanism underlying PD-L1 upregulation in EBV-infected NPC and found that PD-L1 is up-regulated by LMP1-mediated oncogenic pathways and by the excretion of IFN-γ. Our observations here warrant further studies to determine the mechanisms underlying PD-L1 upregulation in LELCC and whether PD-L1 expression can be used to predict clinical response to anti-PD-L1/PD-1 axis immunotherapy.

## MATERIALS AND METHODS

### Tumor specimens and clinical data collection

The study was approved by The Clinical Research Ethics Committee of Fudan University Shanghai Cancer Center and Shanghai Eastern Hepatobiliary Surgery Hospital and was carried out with consent from all patients. We analyzed 13 cases of surgically resected LELCC from the files of Department of Pathology, Fudan University Shanghai Cancer Center and Shanghai Eastern Hepatobiliary Surgery Hospital. All the patients had undergone systemic examination to rule out metastatic tumors. Meanwhile, 15 cases of conventional intrahepatic cholangiocarcinoma (bile duct type) were randomly selected for comparison. All the cases were reviewed by two pathologists and the histological diagnoses were confirmed without discrepancy. Clinical findings, including age, gender, tumor location and size, therapy and clinical outcome were obtained from the medical record, pathology report, or discharge summary. The disease-specific survival (DSS) was defined as the length of time between the surgery and death specifically from this cancer.

### EBV-encoded RNA *in situ* hybridization

EBV-encoded RNA (EBER) *in situ* hybridization was performed with INFORM EBER Probes (a probe used for the detection of early RNA transcript of EBV infection, Catalog number 800-2842, Ventana, Tucson, AZ, USA) and Ventana Medical Systems' ISH *i*VIEW_Blue_ Detection Kit (Catalog number 800-092, Ventana, Tucson, AZ, USA) on 4 μm-thick formalin-fixed, paraffin-embedded sections. The reaction was detected using Ventana Medical Systems' Red CounterstainII (Catalog number 780-2218, Ventana, Tucson, AZ, USA). A case of EBV^+^ nasopharyngeal carcinoma (NPC) was used as a positive control.

### Immunohistochemical staining and evaluation

Immunohistochemical study was performed on 4 μm-thick formalin-fixed, paraffin-embedded sections with an automated immunohistochemical stainer (Ventana, Tucson, AZ, USA). The primary antibodies used in the study included anti-hepatocyte paraffin (HepPar)-1 (Clone OCH1E5, Dako A/S, Denmark), anti-cytokeratin 7 (CK7) (Clone OV-TL 12/30, Dako A/S, Denmark), anti-cytokeratin 19 (CK19) (Clone RCK108, Dako A/S, Denmark) and anti-PD-L1 (Clone SP263, Ventana, Tucson, AZ, USA). Omission of primary antibody and substitution by non-specific immunoglobulins were used as negative controls. The appropriate specificity and sensitivity of the antibody against PD-L1 staining was determined using human placenta as a positive control. Appropriate positive controls were run concurrently for all antibodies tested. Marker stains were coded as positive (staining in more than 5% of cells) or negative (staining in less than 5% of cells). PD-L1 expression showed membranous staining and/or cytoplasmic staining and was divided into weak (scored as 1), moderate (scored as 2) and strong (scored as 3) based on staining intensity. The proportion of immunostained cells was evaluated for tumor cell and tumor-infiltrating immune cells. Patients with at least 5% or greater PD-L1 staining of tumor cells or immune cells were considered positive. At this threshold, PD-L1 expression correlates with response to anti-PD-L1 immunotherapy [43].

### Statistical analysis

Fisher's test was used to test differences between groups. The difference in survival between groups was assessed by the Kaplan-Meier method. Differences were considered significant at *P* < 0.05. SPSS (Chicago, IL, USA) version18.0 was used to analyze all data.
